This article has been retracted.

# Synthesis, characterization, and theoretical studies of the photovoltaic properties of novel reactive azonitrobenzaldehyde derivatives†

**DOI:** 10.1039/d1ra05075c

**Published:** 2021-09-09

**Authors:** Hitler Louis, Izubundu B. Onyebuenyi, Joseph O. Odey, Azuaga T. Igbalagh, MaryJane T. Mbonu, Ededet A. Eno, Anthony M. S. Pembere, Offiong E. Offiong

**Affiliations:** Computational and Bio-Simulation Research Group, Department of Pure and Applied Chemistry, University of Calabar Calabar Nigeria louismuzong@gmail.com shies4me@gmail.com; Department of Pure and Applied Chemistry, Faculty of Physical Sciences, University of Calabar Calabar Nigeria; Department of Chemical Sciences, Federal University of Wukari Wukari Nigeria; Department of Physical Sciences, Jaramogi Oginga Odinga University of Science and Technology Bondo Kenya

## Abstract

All dyes conduct but at different degrees of absorption; it is interesting to study the degree of conductivity and absorptivity of novel reactive azo-dyes in respect to dye-sensitized solar cells (DSSCs) to ascertain their viability for such applications. In this study, four novel reactive azo-dyes were experimentally synthesized from *p*-aminobenzaldehyde, 4-amino-3-nitrobenzaldehyde, and aniline through series of condensation and coupling reactions. The various functional groups, molecular connectivities, and molecular weight of the various fragments of the synthesized dyes were elucidated using the GC-MS, FT-IR, UV-vis, and NMR respectively. The experimentally determined structures were modeled and investigated using density functional theory (DFT) and time-dependent density functional theory (TD-DFT) approaches to computationally compute the electronic structure properties, reactivity, absorption and solvatochromism in four different phases: gas, ethanol, acetone, and water, and the photovoltaic properties for possible applications in dye-sensitized solar cells (DSSCs). By comparing the HOMO (*E*_H_) and the LUMO (*E*_L_) energies from the results obtained demonstrates that dye D has the highest *E*_L_ energy value of −2.48 eV with a relatively lowest *E*_H_ energy value of −5.63 eV such that it lies underneath the conduction band edge of TiO_2_ which is necessary to enable charge regeneration. Pi-electron delocalization was observed from the natural bond orbital (NBO) calculations between the different aromatic rings with dye B and A having the relatively highest and least second-order stabilization energies between σ* → σ* and LP* → LP interacting orbitals respectively. It is also observed in all the solvents that the Gibbs free energy of injection (Δ*G*_inject_) is greater than 0.2 eV and hence, all the studied azo structures in the four phases provided efficient electron injection and light harvesting efficiency (LHE), however, the value of Δ*G*_inject_ for dyes B and D is greatest in all the four phases and thus, provided the highest electron injection of all the dyes. From the fact-findings of quantum theory of atoms-in-molecules (QTAIM), dyes A and C have extra-stability due to their relatively high numbers of intramolecular H-bond interactions along with some additional intra-atomic bonding between atoms within the studied compounds. Hence, all the four dyes are good for DSSCs applications.

## Abstract 2

Four novel reactive azo-dyes were experimentally synthesized from *p*-aminobenzaldehyde, 4-amino-3-nitrobenzaldehyde, and aniline through series of condensation and coupling reactions, and their properties were assessed for possible application in dye-sensitized solar cells.

## 1 Introduction

For decades, extensive research and continuous experiments have shown that dye-sensitized solar cells (DSSCs) have received a lot of attention due to their excellent photovoltaic performance.^1–6^ It can be evidently stated that dye-sensitized solar cells are low cost solar cells based on a semiconductor formed between a photo-sensitized cell and an electrolyte, belonging to a group of thin-film solar cells. Co-invented in 1988 by Brian O'Regan and Michael Grätzel, DSSCs help in converting solar energy to electrical energy.^7^ DSSCs have captivated the minds of researchers due to their numerous advantages which include: low-light performance, optimized performance, high temperature performance, low energy manufacturing process, eco-friendly behavior, ability to be used on variety of substrates, and versatile product integration.^8–11^ Many other future advantages of DSSC are yet to be harnessed which include: coloring, transparency and increases in power density.^9^ In a world where the demand for energy is increasing by the day, and the threat to the environment is becoming alarming, there is a great need to devise environmental friendly sources of energy while meeting the energy demands.

A DSSC typically consists of five components, which are: the molecular dye that absorbs sunlight, a wide band gap semi-conductor (TiO_2_), a redox electrolyte [usually the (I^−^/I_3_^−^) redox couple], a counter electrode (typically a piece of glass coated with platinum) and a porous layer which acts as the anode made from titanium dioxide nanoparticles.^12–16^ The molecular dyes are sensitized by sunlight and electron injection occurs; the excited electrons flow into the conduction band of the semiconductor. The electrons from the TiO_2_, flow to the transparent electrode where they complete the circuit and power the load. After going through the external circuit, they flow back to the electrolyte through the counter electrode. The electrolyte then transports the electrons back to the molecular dye and regenerate the oxidized dye.^17^ It is noteworthy to state that every dye conducts but at different degree of absorption. However, it will be interesting to study the degree of conductivity of our novel dyes in respect to solar voltaic cells to ascertain their viability to such application. The choice of these four dyes is because of their high absorption property to light which is due to their reactive moiety and high molar extinction coefficient which ranges between 1.2 × 10^4^ to 7.6 × 10^4^ L mol^−1^ cm^−1^ as recently reported by Odey and coworkers.^12^ Herein, the synthesis, characterization through spectroscopic investigations (FT-IR, UV/vis, and NMR), DFT, and TD-DFT studies of the photovoltaic performances which includes: short circuit current density (*J*_SC_), light harvesting efficiency (LHE), charge injection efficiency, injection driving force, oxidation potential of the dye at excited and ground states, dye regeneration energy, open circuit voltage (*V*_OC_), and reorganization energy parameters along with detail frontier molecular orbital, natural bond orbital, global reactivity descriptors, density of states, absorption and solvatochromism for the investigation of the HOMO–LUMO energies, second order perturbation energies, structure reactivity, contributions of molecular orbitals, the response to light of the different structures in different phases of media respectively and potential energy distribution analysis (VEDA) of four novel reactive azo dyes were presented.

## 2 Experimental

### 2.1 Synthesis of the dye intermediate (4-amino-3-nitrobenzaldehyde)

About 10 g (0.06 mol) 4-acetalaminobenzaldehyde was added to 25 mL of acetic anhydride and heated to 105 °C and vigorously stirred until it completely dissolved. The solution was then cooled rapidly with an ice bath to 30 °C so as to give fine precipitates of the amine. 4 mL nitric acid and 10 mL acetic anhydride were then mixed carefully and the mixture added drop wise to the already stirred suspension of 4-acetalaminobenzaldehyde at such a rate that the temperature did not rise above 35 °C. After the addition of about 1/3 of the acid, colourless crystals of 4-acetalaminobenzaldehyde diacetate were deposited.^18^ Further addition of the acid made the crystals to dissolve, and towards the end of the addition, the temperature was allowed to rise to about 50 °C. The mixture was then stirred with the temperature still maintained at 50 °C for 15 minutes, and then poured into ice cold water (200 mL). The precipitate of 4-acetalamino-3-nitrobenzaldehyde diacetate was filtered off, washed thoroughly with ethanol, and then with water and dried. Recrystallization from ethanol gave pale yellow leaflets of the diacetate. About 6 g of the diacetate was then added to 20 mL of concentrated HCl and heated on a water bath for 15 minutes, after cooling, 30 mL of water was added and 4-amino-3-nitrobenzaldehyde was precipitated. The precipitate was filtered off, washed with water, and dried. The intermediate was then purified by recrystallization from water to give orange needles of the 4-amino-3-nitrobenzaldehyde. The 4-amino-3-nitrobenzaldehyde was then diazotized and added to acetic acid (24 mL), and water (6 mL). The mixture was heated, and then cooled with stirring to about 12 °C to give a clear solution of the diazonium salt. Cyanuric chloride (1 g, 0.005 mol) was condensed by stirring in 25 mL acetone at a temperature below 5 °C for a period of 1 hour. A neutral solution of 1-naphthol-8-amino-3,6-disulphonic acid (H-acid; 1.7 g, 0.005 mol) in aqueous solution of Na_2_CO_3_ (10% w/v) was added in small amount over a period of 1 hour. The pH was maintained at neutral by simultaneous addition of 30 g Na_2_CO_3_ solution (1% w/v). The reaction mixture was stirred at 0–5 °C for another 4 hours in order to obtain a clear solution; the resulting product was then used directly.

#### 2.1.1 Preparation of dye A

A previously prepared diazonium solution of *p*-aminobenzaldehyde (0.6 g, 0.005 mol) in 5 mL water was added drop wise to an ice cold, well stirred solution of cyanurated H-acid (1.7 g, 0.005 mol) over a period of 10–15 minutes. The pH was maintained at 7.5–8.5 during the addition by simultaneous addition of 10% w/v Na_2_CO_3_. Stirring was then carried out for 4 hours, maintaining the temperature at 5 °C. The mixture was then heated to 60 °C, and NaCl (5 g) was added to the mixture and stirred for an hour. A solid precipitate was formed, which was filtered, and washed with minimum amount of NaCl (5% w/v). The solid was dried at a temperature of 80–90 °C and extracted with dimethlyformaldehyde (DMF). The dye was precipitated by diluting the DMF-extract with excess chloroform; it was filtered, washed with chloroform and dried at 60 °C.

#### 2.1.2 Preparation of dye B

The same coupling conditions and procedures employed in the synthesis of dye A were used, except that a diazonium solution of 4-amino-3-nitrobenzaldehyde was used as the diazo component.

#### 2.1.3 Preparation of dye C

The coupling conditions and procedures employed in the two series of dyes above were used, except that diazotized aniline was used, with cyanurated H-acid.

#### 2.1.4 Preparation of dye D

This series of dyes was synthesized using diazotized *p*-aminobenzaldehyde, except that in this case, non-cyanurated coupling components were used, that is, non-cyanurated H-acid.

### 2.2 Purification of dyes

The synthesized dyes were purified using recrystallization method, by dissolving in ethanol and heating to boiling; the dyes were then quickly filtered with the aid of suction pump to remove insoluble materials, and then allowed to cool down and the crystals were filtered out and dried. The melting points of the purified dyes were determined using the Gallenkamp melting point apparatus.

### 2.3 Infrared spectroscopy of the synthesized dyes

The IR absorption spectra of the dyes were acquired using FTIR-8400S Fourier Transform Infrared Spectrophotometer in order to determine the functional groups present in the newly synthesized reactive dyes.

### 2.4 UV-visible absorption measurements

The UV-visible absorption of the synthesized dyes was carried out at National Research Institute for Chemical Technology (NARICT), Zaria using the V2.30 version of UV-2500PC Series in order to obtain the visible properties of the dyes.

### 2.5 GC-MS spectroscopy of the synthesized dyes

The GC-MS spectroscopy of the synthesized dyes was carried out at National Research Institute for Chemical Technology (NARICT), Zaria using the GC-MS-QP2010 PLUS Series in order to elucidate the molecular weights of the representative dyes.

### 2.6 Schematic routes showing the synthetic pathways

The syntheses of the dyes, diazotization and general reaction routes are shown in Fig. 1 through 6.

#### 2.6.1 Synthesis of dye intermediate

**Fig. 1:** Synthesis of 4-amino-3-nitrobenzaldehyde.

**Fig. 2:** Diazotization of *p*-aminobenzaldehyde.

**Fig. 3:** Diazotization of 4-amino-3-nitrobenzaldehyde.

**Fig. 4:** Diazotization of aniline.

**Fig. 5:** Cyanuration of H-acid.

#### 2.6.2 Diazotization process

#### 2.6.3 Preparation of coupling components

#### 2.6.4 Dye synthesis

**Fig. 6:** General reaction route for the synthesis of the dyes. Where: dye A, “X” = *p*-aminobenzaldehyde, and “R” = cyanurated H-acid. Dye B “X” = 4-amino-3-nitrobenzaldehyde, and “R” = cyanurated H-acid. Dye C “X” = aniline, and “R” = cyanurated H-acid. Dye D, “X” = *p*-aminobenzaldehyde, and “R” = non-cyanurated H-acid.

### 2.7 Computational details

The ground state geometrical structures of the synthesized azo compounds have been modeled and optimized using electronic structure theory based on density functional theory (DFT) and the B3LYP functional with the 6-31+G(d,p) basis set.^19^ The synthesized structures have been co-named as dye A, dye B, dye C and dye D respectively and their structures, FT-IR, GC-MS, UV-vis, and NMR spectra are presented in Fig. S1, S2, S3 through S20 respectively of the ESI.† This DFT computational approach has been widely used in the theoretical investigations of organic dyes for dye-sensitized solar cell applications. Frequency calculations were also done with the same level of theory and none of the frequency calculations generated imaginary frequencies indicating that the optimized geometries are true energy minima. Vertical excitation energy calculations have been done for the first 5 singlet states by using the TD-SCF and long-range CAM-B3LYP/6-31+G(d,p) DFT method in gas, ethanol, acetone, and water media. Electronic excitation energies were determined using the CAM-B3LYP Coulomb-attenuated functional because CAM-B3LYP provides the best overall performance; no correlation is observed between excitation energy errors and reflecting the good quality, balanced description of all categories of excitation energies.^20^ All the computational calculations have been accomplished with density functional theory (DFT) using the Gaussian09W and GaussView6.0.16 suite of programmes.^31^ Surface and structural analysis were carried out with the Multiwfn 3.7 (dev) function analyzer^32^ which can be freely obtained from http://sobereva.com/multiwfn. The NBO computation was conducted using the in-build Gaussian 3.1 method available in Gaussian 09 software.^21^ Pre-geometry optimization using the molecular mechanic optimization with MM + force field implemented in the HyperChem program^22^ has been performed on model structures and outputs used for further geometry optimization at the B3LYP/6-31+G(d,p) level of theory. Natural bond orbital (NBO) analyses were calculated by the NBO 3.1 module embedded in Gaussian. In the calculation, a 6-31+G(d,p) basis set was used for the investigation and using water solvation model as an implicit approach. The Quantum theory of atoms-in-molecules (QTAIM) investigations and all other wavefunction analyses were conducted with the help of Multiwfn 3.7 dev, which is a multifunctional wavefunction analysis program developed by Tian Lu's research group.^23^ The entire vibrational assignments of wave numbers of the various studied compounds were made on the basis of potential energy distribution (PED) by the Vibrational Energy Distribution Analysis (VEDA) 4 program.^24^ Unless otherwise specified, the default settings were used throughout our calculations.

The molecular electronic properties along with the reactivity of the dyes were calculated at the DFT/6-31+(d,p) level of theory by invoking the well-known Koopman's theorem.^25^ The *E*_HOMO_ and *E*_LUMO_ (energies of the HOMO and LUMO orbitals) describe the dyes readiness to undergo electrophilic and nucleophilic attack respectively. There are certain properties the studied dyes must possess to enable them serve as good DSSCs in which TiO_2_ is used as the conduction band. The energy of the LUMO orbital of the dye must lie above the conduction band edge, CBE, of TiO_2_ (−4.0 eV). This is important because fast electron injection from the excited states of the dyes to the TiO_2_ conduction band is beneficial in improving the performance of DSSCs. The energy of the HOMO orbital of the dye must lie below the redox potential of the (*I*^−^/*I*_3_^−^) couple (−4.80 eV), which is necessary to enable charge regeneration of the dyes.^26,27^

Δ*E*_LUMO_ is described as the difference between the energy gap of *E*_LUMO_ of the dyes and *E*_CB_ of TiO_2_. It is mathematically represented as:

1 Δ*E*_L_ = *E*_LUMO_(dye) − *E*_CB_(TiO_2_)

Δ*E*_HOMO_ is described as the difference of *E*_redox_ of (*I*^−^/*I*_3_^−^) and *E*_HOMO_ of the dyes. It is mathematically represented as:

2 Δ*E*_H_ = *E*_redox_(*I*^−^/*I*_3_^−^) − *E*_HOMO_(dye)

Δ*E*_HL_ is described as the energy gap or difference between *E*_HOMO_ and *E*_LUMO_ of the dyes. It is mathematically represented as:

3 Δ*E*_HL_ = *E*_LUMO_ − *E*_HOMO_

According to molecular orbital theory approaches,^28,29^ the HOMO energy (*E*_HOMO_) is related to the ionization potential, IP, and the LUMO energy (*E*_LUMO_) is used to estimate the electron affinity (EA); making it possible to calculate other quantum chemical descriptors such as electron affinity, hardness, softness, electronegativity and electrophilicity index. For DSSC, the IP and EA describe the energy barrier of both holes and electrons. The IP and EA are mathematically represented as:

4 IP = −*E*_HOMO_

5 EA = −*E*_LUMO_

The values of IP and EA are essential for determining the hole–electron donating and accepting ability of both holes and electrons. A low IP is essential for increasing hole-creating ability. A higher EA is important for improving the electron-accepting ability. Using Koopman's theorem for closed shell molecules electronegativity (*χ*), chemical potential (*μ*), hardness (*η*), electrophilicity index (*ω*), electro-accepting power (*ω*^+^) and electro-donating (*ω*^−^) can be redefined as:67891011

The electrochemical potential, *μ* is just the negative of electronegativity. It describes the method of charge transfer in a molecule in its ground state geometry. Chemical hardness (*η*) measures the chemical activity of an element (dye) by determining the resistance to charge transfer in electron number. The chemical reactivity and stability of a molecule (dye) is completely dependent on the chemical hardness of the molecule, which also relates with ICT.^30,31^ The larger the value of chemical hardness the more resist ICT and more stable the compound. Electrophilicity index encompasses the tendency of an electrophile to acquire an extra amount of electron density and the resistance of a molecule (dye) to exchange electron density with the environment. The electron-accepting and electron-donating powers describe the feasibility to accept or accept fractional charges.^32^

## 3 Results and discussion

### 3.1 Structural analysis

#### 3.1.1 FT-IR analysis

The FT-IR spectra of the synthesized compounds in general show some primary characteristics functional groups such as O–H, N–H, and C–Cl present in the dyes as reported in Fig. S2(a)–(d) of the ESI.† The spectra reveals broad band peaks at 3400–3505 cm^−1^ demonstrating the appearance of O–H and N–H stretching vibrations of amino and hydroxyl groups present in the synthesized dyes as well as C–Cl and C–N stretching vibrations of cyanuric chloride at 542–800 cm^−1^ and 1080–1360 cm^−1^ respectively.

Dye A which was experimentally synthesized by using diazotized *p*-aminobenzaldehyde as the diazo component and cyanurated H-acid as the coupling component produce absorption peak due to O–H group at 3422.80 cm^−1^. The carbonyl (C=O) peak was observed at 1639.55 cm^−1^ due to the aldehyde group, SO_3_H peak at 638.46 cm^−1^, N=N stretching at 1483.31 cm^−1^ due to azo group, C–H stretch at 2782.41 cm^−1^, the presence of cyanuric chloride is responsible for C–N and C–Cl peaks respectively at 1174.69 cm^−1^, and 542.02 cm^−1^.

When cyanurated H-acid was used as the coupling component, dye B was obtained with characteristic peaks as follows; O–H at 3428.58 cm^−1^, CHO at 1414.83 cm^−1^, SO_3_H peak at 627.85 cm^−1^, N=N at 1565.29 cm^−1^, C–N at 1193.98 cm^−1^.

Dye C was synthesized using aniline as diazo component, and cyanurated H-acid coupling component. The peak due to O–H group was at 3425.69 cm^−1^, SO_3_H at 615.31 cm^−1^, N=N peak at 1491.99 cm^−1^, C=C stretch at 1402.30 cm^−1^, C–N at 1184.33 cm^−1^, and N–H stretch at 1629.90 cm^−1^.

Dye D was obtained by means of H-acid as the coupling components. The peak due to O–H group in dye D was at 3417.98 cm^−1^, CHO at 1622.19 cm^−1^, SO_3_H at 614.35 cm^−1^, N=N at 1466.91 cm^−1^, C–H at 2797.84 cm^−1^, C=C peak at 1410.98 cm^−1^, C–N at 1181.44 cm^−1^, and N–H stretch at 830.38 cm^−1^.

The spectral assignments along with the potential energy distributions (PED) of all the studied dyes are presented in Table 1.

**Table 1:** Experimental and theoretical spectral assignments and potential energy distribution of the four dyes

S. no.	Dye A		Dye B		Dye C		Dye D		Major vibrations
	Expts	Theory	Expts	Theory	Expts	Theory	Expts	Theory	
1	3422.80	3704.00	3428.58	3632.00	3425.69	3628.00	3417.98	3629.00	*ϑ*_s_OH
2	2782.41	3190.00	2897.33	2910.00	2800.24	2825.00	2797.84	2906.00	*ϑ*_s_CH
3	1639.55	1639.00	1565.29	1581.00	1402.30	1402.00	1410.98	1435.00	*ϑ*_s_CC
4	1174.69	1179.00	1193.98	1217.00	1184.33	1178.00	1181.44	1169.00	*ϑ*_s_NC
5	552.02	558.00	627.85	724.00	615.31	588.00	614.98	655.00	*ϑ*_s_SO
6	1483.31	1448.00	1565.29	1581.00	1491.99	1493.00	1466.91	1304.00	*ϑ*_s_NN

#### 3.1.2 GC-MS analysis

The chromatograms show the composition of the structures of the specimen in suitable solvents (methanol in this experiment) and are a powerful tool for ascertaining the type chemical component that constitutes the dye. For the purpose of interpretation, it is important to note that, the molecular weight of the combined structure of each of the dyes goes well beyond the calibrated range of the GC-MS machine used; hence, the results are segmented. These different segments have to be combined to have a full structure of the samples. Also, the structures obtained are a representation of the chemical composition of the samples under study, providing the basic points and fragments. The GC-MS of the studied dyes gives a complete elucidation of the structure, and from Fig. S3 of the ESI,† the parent mass-to-charge ratio (*m*/*z*) of the different fragment patterns present in the structures are: 27, 28, 41, 46, 270, and 284 corresponding respectively to C_2_H_3_, C_2_H_4_ : CO : H_2_CN, C_3_H_5_ : C_2_H_3_N, NO_2_, C_17_H_34_O_2_, and C_18_H_36_O_2_ species present in the synthesized compounds.

### 3.2 Quantum descriptors (frontier molecular orbital, FMO)

The synthesized reactive dyes were optimized and calculated using four essential solvents based on the experimental conditions and the calculated values for HOMO, LUMO, energy gap, and the global reactivity descriptors of the dyes were carefully studied and presented in Table 1. It is observed that dye C has the highest IP and EA value signifying that dye C is a better acceptor and a bad donor than the other dyes. The HOMO values for the gas phase follows the order – dye C < dye A < dye B < dye D. It can be clearly stated that dye C has the highest HOMO (*E*_H_) value than the corresponding dyes and it lies a bit above the redox potential of the (I^−^/I_3_^−^) couple. The LUMO values for the gas phase follows the order – dye D < dye B < dye A < dye C. Comparing *E*_H_ and *E*_L_, it shows that dye D has the highest *E*_L_ results but the lowest *E*_H_ result so that it lies underneath the conduction band edge of TiO_2_ which is necessary to enable charge regeneration. The values gotten for both *V*_OC_ and *E*_L_ are the same, therefore, the higher the values of *E*_L_, the higher the values of *V*_OC_ also leading to a higher efficiency in DSSC. The band gap values for the gas phase follows the order – dye B < dye D < dye A < dye C. The dye with the least energy gap has a maximum absorption peak, red-shift, and a relatively high light-harvesting efficiency (LHE).

The pattern for the HOMO value for the ethanol phase is dye C > dye A > dye B > dye D. Dye C has the highest HOMO value while dye D has the lowest; for LUMO, the order is dye D > dye B > dye A > dye C, implying that dye D has the highest LUMO value. As for acetone, dye C has the highest HOMO value and follows the decreasing order of dye C > dye A > dye B > dye D; for LUMO, dye B has the highest value and follows the order dye B > dye D > dye A > dye C; and for water phase, dye C has the highest HOMO value and follows the order; dye C > dye A > dye B > dye D, and dye D with a value of 1.34 eV has the highest LUMO value and follows the order; dye D > dye B > dye A > dye C. All the dye sensitizers have well separated HOMO and LUMO energy levels and these results are presented in Table 2 while the energy level diagrams, the optimized structure, and the electrostatic potential structures are displayed in Fig. 7. The dyes get excited by absorbing light of appropriate intensity (sunlight), providing electron injection into the TiO_2_ layer of the dye. Therefore, dyes with a small energy gap (Δ*E*_HL_) have a maximum absorption peak (red-shift) and a relatively high light harvesting efficiency (LHE).^33^

**Table 2:** The quantum descriptors consisting of ionization potential (IP), electron affinity (EA), HOMO and LUMO orbital energies (*E*_H_ and *E*_L_) of the four dyes in gas, ethanol, acetone and water phases

Solvents	Dye	IP	EA	Δ*E*_HL_	Δ*E*_H_	Δ*E*_L_	*η*	−*μ*	*ω*	*ω* ^+^	*ω* ^−^
Gas phase	Dye A	6.08	3.13	2.97	1.28	0.87	1.48	4.61	14.34	5.07	9.68
	Dye B	5.89	2.69	3.20	1.09	1.31	1.60	4.29	11.50	3.81	8.10
	Dye C	6.34	3.42	2.92	1.55	0.57	1.46	4.88	16.31	5.90	10.79
	Dye D	5.63	2.48	3.15	0.83	1.52	1.58	4.06	10.44	3.39	7.44
Ethanol phase	Dye A	5.96	3.01	2.95	1.16	0.99	1.48	−4.49	13.64	4.76	9.25
	Dye B	5.77	2.69	3.08	0.97	1.31	1.54	−4.23	11.62	3.89	8.18
	Dye C	6.06	3.22	2.84	1.26	0.78	1.42	−4.64	15.16	5.44	10.08
	Dye D	5.70	2.65	3.05	0.90	1.35	1.53	−4.18	11.43	3.82	7.99
Acetone phase	Dye A	5.97	3.01	2.96	1.17	0.99	1.48	−4.49	13.62	4.75	9.24
	Dye B	5.72	2.63	3.10	0.92	1.38	1.55	−4.17	11.22	3.72	7.89
	Dye C	6.03	3.16	2.87	1.23	0.84	1.44	−4.60	9.83	5.24	9.83
	Dye D	5.70	2.65	3.05	0.90	1.35	1.53	−4.18	11.43	3.82	7.99
Water phase	Dye A	5.96	3.00	2.96	1.16	1.00	1.48	−4.48	13.56	4.73	9.21
	Dye B	5.78	2.71	3.07	0.98	1.29	1.54	−4.25	11.74	3.94	8.18
	Dye C	6.07	3.23	2.84	1.27	0.77	1.42	−4.65	13.23	5.47	10.12
	Dye D	5.70	2.66	3.04	0.90	1.34	1.52	−4.18	11.50	3.85	8.03

**Fig. 7:** Optimized structure, HOMO, energy levels, LUMO, and electrostatic potential.

### 3.3 Hole–electron analysis

The overlapping integral of the hole–electron distribution can be used to identify a transition mode in a local excitation (LE) and the space between the centroid of the hole and electron is a pointer to the charge transfer of the present transition mode. Some of the hole–electron excitation parameters are; the Sr index which gives the overlap of the electron and hole, the *D* index which gives the overall magnitude of charge transfer length, the *T*-index which measures the separation extent of the hole and electron in charge transfer direction,^12,34^ the *H* index which reflects the breath of the average distribution of hole and electron, the hole delocalization index (HDI), and the electron delocalization index (EDI) are calculated and given in Table 3. In all the studied dyes, dye A has the highest *D* index value with S_0_ → S_2_ and S_0_ → S_3_ having values of 3.30 Å and 3.57 Å therefore referred to as charge transfer, CT excitation. The *D* index follows the pattern; dye A > dye C > dye B > dye D. In the *H* index, the highest excitation value comes from dye C (S_0_ → S_1_, S_0_ → S_3_) and dye D (S_0_ → S_1_, S_0_ → S_3_) respectively but generally all the dyes have high excitation values. Some of the values in the *T* index are positive, indicating splitting of hole and electron. Dye A (S_0_ → S_2_, S_0_ → S_3_) and dye D (S_0_ → S_1_) contain positive values making them CT excitations. It can be observed that the amount of charge transfer in dye A is greater than those in dye D. The negative *T* values signify very low degree of separation of hole and electron.

**Table 3:** The properties of the three excitations for five dyes calculated at TD-SCF/DFT/6-31+G(d)

Dye	Type	*D* (Å)	Sr	*H* (Å)	*T* (Å)	HDI	EDI
Dye A	S_0_ → S_1_	0.29	0.57	2.90	−1.57	15.36	7.65
	S_0_ → S_2_	3.30	0.64	3.53	0.17	7.05	7.76
	S_0_ → S_3_	3.57	0.40	2.57	1.32	23.20	8.13
Dye B	S_0_ → S_1_	0.55	0.54	2.76	−1.52	13.81	8.57
	S_0_ → S_2_	1.07	0.72	3.81	−2.18	6.39	7.15
	S_0_ → S_3_	1.77	0.47	2.31	−0.13	23.22	11.20
Dye C	S_0_ → S_1_	0.68	0.59	3.14	−1.48	11.90	7.52
	S_0_ → S_2_	2.26	0.66	2.70	−0.44	6.77	7.71
	S_0_ → S_3_	2.86	0.61	3.99	−0.19	5.47	6.77
Dye D	S_0_ → S_1_	2.16	0.62	3.17	0.19	6.71	9.65
	S_0_ → S_2_	0.53	0.62	2.99	−1.55	10.46	9.80
	S_0_ → S_3_	0.31	0.72	3.52	−1.81	6.12	8.98

### 3.4 Photovoltaic properties

The open circuit voltage (*V*_OC_) is defined as the energy difference between the redox potential of the electrolyte's redox couple (*I*^−^/*I*_3_^−^) and the quasi-Fermi level of the semiconductor's conduction band (TiO_2_). It is mathematically represented as:12where, *E*_CB_ is the conduction band edge of TiO_2_, *q* is the unit charge, *T* is the absolute temperature, *k* is the Boltzmann constant, *n*_c_ is the number of electrons in the conduction band, *N*_CB_ is the density of accessible states in the conduction band and *E*_redox_ is the redox potential of the electrolyte. ΔCB is the shift of CB when the dyes are adsorbed. It is mathematically represented as:13where *μ*_normal_ is the dipole moment of the individual dye molecule perpendicular to the surface of TiO_2_, and *γ* is the dye surface concentration, *ε*_0_ and *ε* are the vacuum permittivity and dielectric permittivity respectively. The calculation of *V*_OC_ can also be approximately obtained by the difference between *E*_LUMO_ and *E*_CB_. It is used for this purpose because the studied dyes are singly not in the adsorbed state on TiO_2_. Therefore, calculations of *n*_c_ and *N*_CB_.

*J*_SC_ can be mathematically represented as:14LHE (*λ*) is the light harvesting efficiency at maximum wavelength, *ϕ*_inject_ is the electron injection efficiency, and *η*_collect_ is the charge collection efficiency. To obtain a high *J*_SC_, LHE and *ϕ*_inject_ should be as high as possible. The LHE can be mathematically expressed as:

15 LHE = 1 − 10^−*f*^

where *f* is the oscillator strength of the dye corresponding to *λ*_max_, *ϕ*_inject_ is related to the thermodynamic driving force Δ*G*_inject_ of electron injection from the excited states of dye to conductive band TiO_2_

Δ*G*_inject_ (the free energy difference for electron injection) is mathematically represented as:16where *E*^dye*^ is the redox potential of the oxidized dye at excited state. *E*^dye^ is the redox potential of the oxidized dye at ground state and Δ*E* is the lowest vertical excitation energy.  is the energy of the conductive band edge of TiO_2_.

Δ*G*_reg_ (the driving force for dye regeneration) is mathematically represented as:

17 Δ*G*_reg_ = *μ*(*I*^−^/*I*_3_^−^) − *E*^dye^

A value of Δ*G*_reg_ greater than 0.2 eV for an oxidized dye could be the efficient electron injection.^35^ In order to determine the value of *J*_SC_ and the overall conversion efficiency (*μ*), the calculated values of *V*_OC_, *f*, LHE, *λ*_max_, Δ*G*_inj_, Δ*G*_reg_, Δ*G*_cr_ in four different solvents along with the changes in wavelength are reported in Table 4. From eqn (12) it is observed that a dye with a small energy band gap is beneficial to a red-shifted absorption spectrum and gives rise to more electrons corresponding to an increase in *n*_c_ and thus, increases the efficiency of *V*_OC_. In calculating Δ*G*_reg_, it is important to note that the experimental value of *E*_CB_ used for the TiO_2_ semiconductor is −4.00 eV.^36,37^ It is observed that in all the solvents Δ*G*_inject_ is greater than 0.2 eV and therefore, all the dyes in the four phases provide efficient electron injection, however, the value of Δ*G*_inject_ for dyes B and D is greatest in all the four phases and thus, provide the highest electron injection of all the dyes. It is also observed that the Δ*G*_reg_ for all the dyes in the four phases is less than 0.4 eV and hence, the dyes have low or no effect on Δ*G*_reg_. The results in Table 4 also shows that among the studied dyes in the four phases the highest values of *f* come from dyes B and D, but the value of LHE varies and shows greater stability in dyes B and D. Dyes B and D still possess the highest value of *V*_OC_ in all studied phases.

**Table 4:** Photovoltaic properties of the four dyes in gas, ethanol, acetone and water phases

Solvent	Dye	*V*_OC_	*f*	LHE	*λ*_max_ (eV)	Δ*G*_inj_	Δ*G*_reg_	Δ*G*_CR_
Gas phase	Dye A	0.87	0.34	0.54	3.35	1.17	−1.67	4.12
	Dye B	1.31	0.81	0.85	3.54	1.36	−2.11	4.56
	Dye C	0.57	0.34	0.54	2.56	0.91	−1.37	3.82
	Dye D	1.52	0.43	0.63	2.97	1.62	−2.32	4.77
Ethanol phase	Dye A	0.99	0.40	0.60	2.55	1.29	−1.79	4.24
	Dye B	1.31	0.87	0.87	3.34	1.48	−2.11	4.56
	Dye C	0.78	0.37	0.57	2.42	1.19	−1.58	4.03
	Dye D	1.34	0.50	0.56	3.49	1.55	−2.14	4.59
Acetone phase	Dye A	0.99	0.39	0.59	2.55	1.28	−1.79	4.24
	Dye B	1.38	0.87	0.87	3.37	1.53	−2.18	4.63
	Dye C	0.84	0.36	0.87	2.45	1.22	−1.64	4.09
	Dye D	1.35	0.52	0.86	3.51	1.55	−2.15	4.60
Water phase	Dye A	1.00	0.39	0.59	2.55	1.29	−1.80	4.25
	Dye B	1.29	0.85	0.86	3.34	1.47	−2.09	4.54
	Dye C	0.77	0.36	0.56	2.41	1.18	−1.57	4.02
	Dye D	1.35	0.53	0.71	3.51	1.55	−2.15	4.60

### 3.5 Quantum theory of atoms in molecules (QTAIM)

The Multifunctional analyzer dev 2.7 was used for the investigation of the quantum theory of atom-in-molecules (QTAIM) which is the most popular theory for investigation of H-bonds at electronic structure level.^38,39^ Intramolecular H-bond is one of the most notable features which could affect relative stability and reactivity among the various studied compounds. In this theory, critical points are the positions where gradient of electron density *ρ* is zero, which can be further classified according to the sign of eigenvalues of Hessian matrix of *ρ*. Bond critical points (BCP) have two negative eigenvalues; they usually occur between interacting atom pairs, and real-space properties at a BCP have a close relationship with the natural and strength of the interaction. Under the AIM framework, Lipkowski *et al.*,^40^ proposed three criteria for existence of H-bond: (1) The H-bond must be accompanied by a BCP; (2) *ρ* at BCP (*ρ*_BCP_) should be within 0.002–0.04 a.u.; and (3) ∇^2^*ρ* at BCP (∇^2^*ρ*_BCP_) should be between 0.02–0.15. The various parameters obtained at the BCP are presented in Table 5. We observed that dye A, in addition to other intra-atomic bond, there are 3 intramolecular H-bonds having electron densities of 0.009, 0.01, and 0.039 corresponding to H-bonds involving C_24_–H_26_⋯O_43_, C_5_–H_10_⋯O_45,_ and O_45_–H_47_⋯N_13_ bonds while the Laplacian of the electron densities associated with such H-bonds are 0.034, 0.044, and 0.087 respectively. In like manner 2 intramolecular H-bonding were revealed for dye B involving O_34_–H_35_⋯N_26_ and C_9_–H_7_⋯O_48_ with corresponding electron densities of 0.04 and 0.011 respectively. Similarly, 2 H-bonds were noticed in dye C having electron density values of 0.009 and 0.004 corresponding to hydrogen interactions of C_20_–H_22_⋯O_28_ and C_2_–H_8_⋯O_25_ bonds respectively. However, dye D is observed to have a single intramolecular H-bonds having electron and Laplacian electron densities of 0.009 and 0.0338 respectively. Hence, dyes A and C are expected to have extra-stability due to their relatively high H-bond interactions along with some intra-atomic bonds.^41^ Because stability is a problem in the photovoltaic application of organic compounds, this extra-stability as a result of intramolecular H-bonds is essential for effective application of the structures in dye-sensitized solar cells.

**Table 5:** Intramolecular H-bonds in the fours dyes A, B, C, and D

Dyes	Interaction	BCP	*ρ*(*r*)	*G*(*r*)	*K*(*r*)	*V*(*r*)	*H*(*r*)	∇^2^*ρ*(*r*)
A	O_27_–H_35_⋯N_12_	70	0.0797	0.0534	0.0224	−0.0758	−0.0224	0.1240
	C_24_–H_26_⋯O_43_	106	0.0089	0.0071	−0.0014	−0.0056	0.00143	0.0340
	C_5_–H_10_⋯O_45_	77	0.0107	0.0093	−0.0019	−0.0074	0.00193	0.0448
	O_45_–H_47_⋯N_13_	78	0.0393	0.0237	0.0021	−0.0259	−0.0021	0.0866
	O_27_⋯N_28_	80	0.0160	0.0134	−0.0012	−0.0122	0.00124	0.0586
B	O_34_–H_35_⋯N_26_	104	0.0402	0.0305	0.0028	−0.0334	−0.0028	0.1110
	C_2_–H_8_⋯O_41_	60	0.2790	0.0338	0.2820	−0.3166	−0.2828	−0.996
	C_9_–H_7_⋯O_48_	54	0.0109	0.0087	−0.0009	−0.0077	0.0009	0.0385
	O_45_–N_28_	61	0.0167	0.0136	−0.0009	−0.0126	0.0009	0.0585
C	C_20_–H_22_⋯O_28_	78	0.0099	0.0078	−0.0010	−0.0068	0.0010	0.0354
	C_2_–H_8_⋯O_25_	110	0.0048	0.0036	−0.0009	−0.0027	0.0009	0.0183
	O_49_–H_50_⋯N_29_	75	0.0604	0.0457	0.0067	−0.0525	−0.0067	0.1562
	O_48_⋯N_29_	68	0.0179	0.0145	−0.0012	−0.0132	0.0012	0.0634
	O_25_⋯N_30_	109	0.0078	0.0060	−0.0006	−0.0054	0.0006	0.0268
	C_38_⋯O_49_	65	0.0148	0.0125	−0.0014	−0.0110	0.0014	0.0557
D	O_24_–H_35_⋯N_35_	46	0.0521	0.0392	0.0051	−0.0443	−0.0051	0.1365
	C_21_–H_23_⋯O_30_	47	0.0095	0.0074	−0.0010	−0.0064	0.00100	0.0338
	O_240_⋯N_31_	58	0.0166	0.0138	−0.0011	−0.0127	0.00111	0.0601

### 3.6 Natural bond orbital (NBO) analysis

The study of natural bond orbital analysis has been performed in this study to chemically understand the nature and type of interaction existing between the Lewis and non-Lewis orbitals of the studied dye molecules, this interaction is noted in terms of charge exchange and conjugative interaction between donor and acceptor orbitals. This analysis is carried out by considering the changes in energy of interaction between donors and acceptor orbital reported as second order perturbation energy obtained from the second order perturbation theory of Fock matrix. The donor–acceptor NBO interaction energy or stabilization energy (*E*^2^) between the orbitals under consideration has been evaluated using eqn (18)18where, *q*_*i*_, *ε*_*i*_, *ε*_*j*_ and *F*(*i*,*j*) are the Lewis (donor) orbital occupancy, *i*^th^ diagonal element, *j*^th^ diagonal element and the off-diagonal NBO Fock matrix element, respectively.

The NBO analysis was calculated at the same level of theory as the optimized structures with the aim of explaining the inter and intra-molecular hydrogen bonding and π electron delocalization within the molecule.^42,43^ Several interactions have been observed in the second order perturbation result reported in Table 6 as well as Tables S1–S4 of the ESI† as bonding, non-bonding and anti-bonding interactions with different respective energies depending on the strength of interaction. The notable and highest interactions result from lone pair to anti-bonding lone pair on carbon and hetero atoms respectively which are classified as non-bonding interactions and have been reported to enhance the stability of molecules.^44–48^ The interaction between lone pair bonding orbital LPO_27_ and anti-bonding lone pair orbital LP*H_35_ has a strong stabilization energy of 379.20 kcal mol^−1^, similarly the interaction of donor orbital LPC_14_ with the anti-bonding orbital π*N_12_–N_13_, and anti-bonding orbital LP*C_15_ with LPC_16_ have remarkable stabilization of 127.60 kcal mol^−1^ and 1726.93 kcal mol^−1^ respectively which signifies the intermolecular charge transfer within the respective molecular fragment; pi-electron delocalization was observed between the different aromatic rings with substantial stabilization energy; such donor and acceptor interactions between the πC_18_–C_19_ and n*C_17_ with a stabilization of 40.05 kcal mol^−1^ and πC_2_–C_3_ and π*C_1_–C_6_ whose stabilization energy is 20.20 kcal mol^−1^ suggests the presence of strong resonance stabilization by pi-electron delocalization which explains the charge transfer or hyper conjugative interaction of Lewis orbital (donor) and non-Lewis orbital (acceptor), the intra molecular hydrogen bonding and delocalization of π electron of the molecule.

**Table 6:** Highest second order perturbation energies of the fours dyes A, B, C, and D

Dye	Donor NBO (*i*)	Acceptor NBO (*j*)	*E*(2), kcal mol^−1^	*E*(*j*) − *E*(*i*), a.u.	*F*(*i*,*j*), a.u.
A	LP*(1) C_15_	LP(1) C_16_	1726.93	0.01	0.131
B	σ*C_19_–C_20_	σ*C_19_–H_44_	64 601.60	0.22	3.399
C	LP*(1) C_3_	LP (1) C_2_	2127.87	0.01	0.139
D	LP(1) C_14_	LP*(1) C_13_	1747.32	0.01	0.132

### 3.7 UV/vis absorption and solvatochromism

The photovoltaic property of dye for DSSCs is used in accessing UV-vis absorption spectrum.^49^ A dye having high efficiency must possess a strong and broad absorption band over the visible light (400–800 nm).^50^ The optimized absorption spectra for the UV-vis in the gas, water, acetone and ethanol phases are displayed in Fig. S4† and their values are listed in Table 7, respectively. Among the studied dyes, the dye with the highest intensity of absorption peak in the gas phase is dye B, signifying its efficiency in the absorption of most photons than the other dyes. The maximum order of the absorption wavelength for the dyes is consistent with the order of the energy gaps, which is to say that the more the red shift of the UV-vis absorption, the narrower the energy gap. Dyes A and C have the same absorption peak value at 510.5 nm. In the acetone phase, the dye with the highest absorption peak is dye B. Dye B also has the highest absorption peak in ethanol and water phases. Wave-length for the dyes is consistent with the order of the energy gap that is to say the more the red shift of the UV-vis absorption, the narrower the energy gap implying that the more polar the solvent the narrower the band gap. Again, the theoretical and experimental UV results are presented in Tables 8 and 9 showing that the values are closely similar in the various solvents except in the case of water which varies a bit higher in the theoretical results when compared with the experimental values.

**Table 7:** Tabulated absorption wavelengths (nm) and major contribution with oscillator strength for the studied dyes in their acetone, ethanol, gas and water phases

Excitation	Wavelength (nm)	Energy (eV)	Oscillator strength	Major contribution (%)	Assignment
**Dye A**					
*Acetone*					
S0 → S1	505.81	2.4512	0.355	H → L (96.24%)	π → π*
S0 → S2	489.65	2.5321	0.054	H−1 → L (57.73%)	n → π*
S0 → S3	400.52	3.0956	0.079	H → L+1 (72.17%)	n → π*
*Ethanol*					
S0 → S1	512.85	2.4175	0.368	H → L (97.47%)	π → π*
S0 → S2	491.97	2.5202	0.040	H−1 → L (59.78%)	n → π*
S0 → S3	410.24	3.0222	0.040	H → L+1 (87.51%)	n → π*
*Gas*					
S0 → S1	495.50	2.5022	0.018	H−1 → L (70.16%)	π → π*
S0 → S2	483.66	2.5635	0.322	H → L (79.89%)	n → π*
S0 → S3	385.25	3.2183	0.255	H−2 → L (58.31%)	n → π*
*Water*					
S0 → S1	515.17	2.4067	0.358	H → L (97.53%)	π → π*
S0 → S2	492.24	2.9931	0.040	H−1 → L (58.25%)	n → π*
S0 → S3	414.23	2.9931	0.040	H → L+1 (89.27%)	n → π*

**Dye B**					
*Acetone*					
S0 → S1	487.31	2.5443	0.0598	H → L (96.24%)	π → π*
S0 → S4	314.97	3.9364	0.3518	H−1 → L (58.81%)	n → π*
S0 → S5	292.48	4.2391	0.4152	H → L+2 (65.99%)	n → π*
*Ethanol*					
S0 → S2	371.59	3.3412	0.8708	H → L (69.83%)	
S0 → S4	315.84	3.9255	0.3740	H−1 → L (62.76%)	
S0 → S5	292.01	4.2459	0.3993	H → L (67.87%)	
*Gas*					
S0 → S2	349.76	3.5449	0.8057	H → L (69.49%)	n → π*
S0 → S4	311.85	3.9757	0.0836	H−2 → L (30.31%)	n → π*
S0 → S5	294.23	4.2139	0.6149	H → L+2 (38.79%)	π → π*
*Water*					
S0 → S2	371.74	3.3353	0.8537	H → L (69.78)	
S0 → S3	314.86	3.9377	0.0022	H−1 → L (63.91)	
S0 → S5	291.28	4.2565	0.3891	H → L+2 (67.87)	

**Dye C**					
*Acetone*					
S0 → S1	505.81	2.4512	0.3558	H → L (96.24%)	π → π*
S0 → S2	489.65	2.5321	0.0543	H−1 → L (57.73%)	n → π*
S0 → S3	400.52	3.0956	0.0791	H → L+1 (72.17%)	n → π*
*Ethanol*					
S0 → S1	512.85	2.4175	0.3686	H → L (97.47%)	π → π*
S0 → S2	491.97	2.5202	0.0430	H−1 → L (59.78%)	n → π*
S0 → S3	410.24	3.0222	0.0403	H → L+1 (87.51%)	n → π*
*Gas*					
S0 → S1	495.50	2.5022	0.0187	H−1 → L (70.06%)	π → π*
S0 → S2	483.66	2.5635	0.3228	H → L (79.89%)	n → π*
S0 → S3	385.25	3.2183	0.2550	H−2 → L (58.31%)	n → π*
*Water*					
S0 → S1	515.17	2.4067	0.3587	H → L (97.53%)	π → π*
S0 → S2	492.24	2.5188	0.0407	H → L (58.25%)	n → π*
S0 → S3	414.23	2.9931	0.0409	H → L+1 (89.27%)	n → π*

**Dye D**					
*Acetone*					
S0 → S1	542.60	2.2850	0.1455	H−1 → L (59.79%)	π → π*
S0 → S2	450.68	2.7510	0.4527	H → L (65.39%)	n → π*
S0 → S3	353.24	3.5099	0.5240	H−2 → L (83.44%)	n → π*
*Ethanol*					
S0 → S1	542.49	2.2855	0.1463	H−1 → L (59.88%)	π → π*
S0 → S2	451.08	2.7486	0.4517	H → L (65.55%)	n → π*
S0 → S3	353.39	3.5084	0.5260	H−3 → L (83.67%)	n → π*
*Gas*					
S0 → S1	552.60	2.2437	0.0786	H → L (46.63%)	π → π*
S0 → S2	417.84	2.9673	0.4323	H−1 → L (48.92%)	n → π*
S0 → S3	368.22	3.3672	0.0003	H−3 → L (83.67%)	n → π*
*Water*					
S0 → S1	541.76	2.2886	0.1450	H−1 → L (60.48%)	π → π*
S0 → S2	451.84	2.7440	0.4426	H → L (66.30%)	n → π*
S0 → S3	353.63	3.5060	0.5259	H−3 → L (84.02%)	n → π*

**Table 8:** Theoretical UV-vis data for the four dyes in different solvents

Dyes	Acetone	Ethanol	Gas	Water
A	505.81	512.85	495.50	515.17
B	487.31	371.59	349.76	371.74
C	505.81	512.85	495.50	515.17
D	542.49	552.60	552.60	541.76

**Table 9:** Experimental UV-vis data for the four dyes in different solvents

Dyes	Acetone	Ethanol	Gas	Water
A	560.00	480.00	—	498.00
B	488.00	403.00	—	400.00
C	512.00	496.00	—	456.00
D	490.00	560.00	—	524.00

### 3.8 Density of states (DOS)

Density of state (DOS) is an important tool in science that helps to facilitate the property of materials. It is made up of conduction bands and surface valence divided by a wide band gap.^51,52^ A resulting DOS graph plot is an important tool for classifying orbital compositions visually when the discrete energy levels are artificially curve broadened. A graph of total DOS (TDOS) map, partial DOS (PDOS) map, and OPDOS map of the four dyes with the help from different sets of molecular orbital was plotted using multi-wave function as displayed in Fig. 8. The TDOS and PDOS axes are at the left hand side while OPDOS are at the right. Oxygen atom fragment attains height of about 0.40 and 0.18 a.u resulting from the highest and lowest energies as seen in dye C and dye A. The nitrogen atom fragment is seen to possess the highest and lowest values at 0.21 and 0.07 a.u in dye A and dye D respectively. The maximum and minimum energies in sulfur are confirmed at 0.19 and 0.12 a.u of dye A and dye B respectively. As for chlorine fragment, the dyes A, B and C are equivalent with a value of 0.24 a.u. The highest and lowest value for carbon fragment is 0.40 and 0.31 a.u from dye B and dye D respectively. The OPDOS present in dye C and dye D with values of −0.10 and 0.01 showing the anti-bonding due to poor overlapping in orbital phase.

**Fig. 8:** Graphical representation of DOS and PDOS for dyes A, B, C and D.

## 4 Conclusion

Four reactive azo dyes were synthesized, spectroscopically investigated along with elucidating the pattern of wavelength absorption in four different solvents. The experimentally synthesized structures were further computationally modeled by means of first principle density functional theory at the B3LYP/6-31+(d,p) method to investigate the ground state electronic structural properties, reactivities, and bonding nature while the excited state molecular properties along with the photovoltaic application of the reactive dyes have been extensively studied using the time-dependent density functional theory (TD-DFT) by imploring the CAM-B3LYP method with 6-311+G(d,p) basis set. The fact-findings reveals that the HOMO and LUMO levels of all the investigated dyes are situated within the I/I_3_^−^ electrolyte and semi-conductor band (TiO_2_) limit respectively. From the extracted values for EA, IP, *ω*^+^ and *ω*^−^, dye C is the best dye in all phases and dye D is the least appropriate dye for DSSCs. From the comparison of *E*_H_ and *E*_L_, it shows that dye D has the highest *E*_L_ but lowest *E*_H_ results such that it lies underneath the conduction band edge of TiO_2_ which is necessary to enable charge regeneration. It is also observed that in all the solvents Δ*G*_inject_ is greater than 0.2 eV. Therefore, all the dyes in the four phases provide efficient electron injection and light harvesting efficiency, LHE; but the value of Δ*G*_inject_ for dyes B and D is greatest in all the four phases and thus, provide the highest electron injection of all the dyes. Dyes A and C have extra-stability due to their relatively high H-bond interactions along with some intra-atomic bonds from the QTAIM results. It can be concluded that Dye B has the highest *E*_HL_ and the highest LHE; dye C has the lowest *E*_HL_ and the lowest LHE along with dye A. Hence, all the four dyes are good for DSSCs applications.

## Funding

This research did not receive funding from any source.

## Authors' contributions

Hitler Louis: conceptualization, design, software, and supervision. MaryJane T. Mbonu: analysis, writing, and manuscript draft. Izubundu B. Onyebuenyi: visualization, writing, and editing. Odey: methodology, validation, and editing. Azuaga T. Igbalagh: methodology and data curation. Ededet A. Eno: validation, visualization, reading, writing, editing. Anthony M. S. Pembere: reading, writing, and editing. Offiong E. Offiong: project administration, validation, visualization, and supervision.

## Conflicts of interest

We declare no conflict of any sort.

## Supplementary Material

RA-011-D1RA05075C-s001
